The article "Serum Vitamin D Level and Efficacy of Vitamin D Supplementation in Children with Atopic Dermatitis: A Systematic Review and Meta-analysis" was published in 2022. Journal: Comput Math Methods Med.

# Serum Vitamin D Level and Efficacy of Vitamin D Supplementation in Children with Atopic Dermatitis: A Systematic Review and Meta-analysis

**DOI:** 10.1155/2022/9407888

**Published:** 2022-07-20

**Authors:** Hongbo Fu, Yanting Li, Huimin Huang, Dan Wang

**Affiliations:** ^1^Department of Emergency, Haikou Maternal and Child Health Hospital, Haikou, 570203 Hainan, China; ^2^Department of Pediatrics, Sanya Traditional Chinese Medicine Hospital, Sanya, 572000 Hainan, China; ^3^Department of Pediatrics, The First Affiliated Hospital of Hainan Medical University, Haikou, 570102 Hainan, China

## Abstract

**Background:**

The relationship between vitamin D and atopic dermatitis (AD) is controversial. This meta-analysis is aimed at exploring vitamin D level and its deficiency in pediatric AD and at evaluating the efficacy of vitamin D supplementation.

**Methods:**

PubMed, Medline, Embase, Ovid, Cochrane Library, ISI Web of Science, and ClinicalTrials were searched. Binary variables and continuous variables were measured by odds ratio (OR) and mean difference (MD) with 95% confidence intervals, respectively. The modified Jadad scale, Newcastle-Ottawa Scale (NOS), and Cochrane's bias risk tools were used to evaluate study quality and the risk of bias of eligible studies, respectively.

**Results:**

A total of 22 literature were included in the analysis. Serum 25 (OH) D level in pediatric AD patients was significantly lower than that of the control group with a combined MD value of -8.18 (95% CI: -13.15, -3.22). Patients with AD were more prone to develop vitamin D deficiency with a combined OR value of 2.17 (95% CI: 1.15, 4.11). According to the score of SCORAD, the level of serum 25 (OH) D level in patients with severe AD was significantly lower than that in patients with mild AD (combined MD = 9.23, 95% CI: 6.92, 11.55). Both self-control studies and randomized controlled trials showed improved SCORAD score and EASI score after vitamin D supplementation.

**Conclusion:**

This meta-analysis showed lower serum 25 (OH) D level and increased risk of vitamin D deficiency in pediatric AD patients as compared with healthy controls. The serum 25 (OH) D level in severe AD patients was significantly lower than that in the mild AD patients. The SCORAD and EASI score improved after vitamin D supplementation, suggesting its beneficial effect to AD patients. At the same time, more homogeneous studies are needed to reduce confounding factors and further evaluate the impact of vitamin D treatment on the outcome of AD patients.

## 1. Introduction

Atopic dermatitis (AD) is a common chronic and recurrent inflammatory skin disease characterized by pruritus, eczema, and dry skin [1]. Usually, AD represents an allergy to allergens and thus is often accompanied by various other allergic diseases, such as allergic asthma or rhinitis [2]. AD is seen predominantly in children, of which 30% will continue into adulthood [3]. As a common disease, it affects 5%-20% of children globally. The incidence rate of AD gradually rises within the time range, especially in countries with high urbanization rates or high latitude regions in winter [4]. The occurrence of AD is mainly the result of epidermal barrier defects and immune disorders, while bacterial and viral infections such as Staphylococcus aureus or herpes simplex virus will aggravate AD [5]. Traditional drugs for AD treatment are antihistamines and immunomodulators that reduce skin inflammation, such as local or oral corticosteroids or calcineurin inhibitors [6]. However, these medications are limited by considerable side effects and poor patient compliance.

The article "Serum Vitamin D Level and Efficacy of Vitamin D Supplementation in Children with Atopic Dermatitis: A Systematic Review and Meta-analysis" was published in 2022. Journal: Comput Math Methods Med.

Currently, a host of studies have reported the potential role of vitamin deficiency in AD development. For example, AD deteriorates in winter when the serum 25 (OH) D level is the lowest [7]. In addition, it was found that the AD symptoms improved after vitamin D supplementation [8]. These studies may also suggest that vitamin D supplementation is a safe and effective alternative therapy for AD. Although several prior investigations have analyzed the relationship between vitamin D and AD, they were limited by a small number of literatures included, low study quality, remote time frame, and mixed results with both children and adult patients included. Currently, there are still debates in terms of the relationship between vitamin D and atopic dermatitis. In addition, effective treatment and unified research conclusions for AD are still lacking [9–11].

We conducted systematic review and meta-analysis of the included literature to determine serum 25 (OH) D levels in pediatric AD patients and explored the relationship between vitamin D deficiency and AD. We also analyzed the relationship between the grading of AD symptoms and serum 25 (OH) D levels by atopic dermatitis index (SCORAD). Finally, we evaluated the effect and efficacy of vitamin D supplementation on AD severity by SCORAD and eczema area and severity index (EASI).

## 2. Methods

### 2.1. Literature Retrieval Strategy

The following databases were searched: PubMed, Medline, Embase, Ovid, Cochrane Library, ISI Web of Science, and ClinicalTrials. The search keywords were “pediatrics” or “children” and “calciferol” and “atopic dermatitis” or “eczema.” The search for the literature was limited to human research. The search process was in accordance with the PRISMA statement, and differences in the process were resolved by negotiation. The literature retrieval time is up to February 2022.

The article "Serum Vitamin D Level and Efficacy of Vitamin D Supplementation in Children with Atopic Dermatitis: A Systematic Review and Meta-analysis" was published in 2022. Journal: Comput Math Methods Med.

### 2.2. Literature Selection

The inclusion criteria were as follows: (1) case-control study or intervention study, including randomized controlled trial (RCT) and self-controlled stud; (2) pediatric AD patients (<18 years old); (3) available data with regard to serum 25 (OH) D levels in patients and control groups, the number of patients with vitamin D deficiency in patients and control groups, the classification of AD symptoms and corresponding serum 25 (OH) D levels; (4) quantitative assessment of the severity of AD by using SCORAD index or EASI score; and (6) the modified Jadad scale score ≥ 4 for RCTs or the Newcastle Ottawa mean scale (NOS) score of ≥7 for a case-control study.

The exclusion criteria were as follows: (1) The types of literature which were review, systematic evaluation, meta-analysis, case report, and editorial article; (2) incorporation of adult (age > 18 years) AD patients; (3) non-English literature; and (4) studies of pregnant women, infants (<1 year old), or umbilical cord blood samples which were included.

### 2.3. Data Extraction

Data were extracted from all literature by two independent authors and recorded in the corresponding tables. The extracted data and characteristics include the following: literature characteristics (author, year of publication, and study design), patient characteristics (age, serum 25 (OH) D level (ng/mL), SCORAD index, or EASI score), degree of vitamin D deficiency, and dose and timing of vitamin D supplementation.

The SCORAD is the most effective and commonly used method to evaluate the prevalence of AD in clinical research [12]. The severity of AD is divided into mild AD with SCORAD < 25, moderate AD with SCORAD > 25, and severe AD with SCORAD > 50.

According to the seven-level classification of international vitamin D nutritional status [13], a serum 25 (OH) D level < 20 ng/mL was defined as vitamin D deficiency.

### 2.4. Study Quality Evaluation

The modified Jadad scale, NOS, and Cochrane's risk of bias tool were employed to assess study quality, bias, and risk of eligible studies, respectively [14]. The modified Jadad scale includes random sequence generation (2 points), randomized hiding (2 points), blinding method (2 points), and withdrawal and dropout (1 point), with a total of 7 points. Studies with 1-3 points were deemed to be of low quality, whereas 4-7points were considered to be high-quality. The NOS scoring table includes the selection of objects in the case combination control group (4 points), the comparability of cases and controls (2 points), and the measurement of exposure factors (3 points), with a total of 9 points. The potential study biases were assessed using Cochrane's bias risk tool in accordance with the PRISMA statement, and the map of the risk of bias was generated [15].

The article "Serum Vitamin D Level and Efficacy of Vitamin D Supplementation in Children with Atopic Dermatitis: A Systematic Review and Meta-analysis" was published in 2022. Journal: Comput Math Methods Med.

### 2.5. Statistical Analysis

Review Manager software was used for establishing a forest map and funnel map. Binary variables and continuous variables were measured by odds ratio (OR) and mean difference (MD), respectively. 95% confidence intervals were used for each variable. Clinically homogeneous studies were divided into subgroups, and meta-analyses were performed accordingly. Heterogeneity testing was done by a chi-square test. The fixed effects model was used when the homogeneity was low (*I*^2^ < 50%). Otherwise, the random effects model was used. When *P* < 0.05, the difference was considered statistically significant.

## 3. Results

### 3.1. Retrieval Results and Literature Quality Evaluation

The process of literature search and screening is shown in Figure 1. A total of 2464 literatures about vitamin D and AD in children were retrieved from the database. After screening according to the inclusion and exclusion criteria, 22 literatures were included in the analysis [16–37], and the basic characteristics and corresponding scores for each document were counted. The diagram of risk of bias for RCTs is shown in Figure 2. The basic characteristics and document quality scores of included documents are shown in Table 1.

### 3.2. Comparison of Serum 25 (OH) D Levels between AD Patients and Healthy Controls

14 studies evaluated the comparison of serum 25 (OH) D levels between AD patients and healthy controls. The characteristics of the included literature are shown in Table 2. A total of 1450 patients and 1009 healthy controls were included. Significant interstudy heterogeneity (*P* < 0.00001, *I*^2^ = 98%) were noted, for which the random effects model was used. The combined MD value was -8.18 (95% CI: -13.15, -3.22), and the combined effects amount was *Z* = 3.23 (*P* = 0.001). The results showed that serum 25 (OH) D level in AD patients was significantly lower than those in healthy controls (Figure 3).

### 3.3. Comparison of Serum 25 (OH) D Deficiency between AD Patients and Healthy Controls

Comparisons of serum 25 (OH) D deficiency between AD patients and healthy controls were reported in 9 studies that included 1096 patients and 765 healthy controls. Significant literature heterogeneity (*P* < 0.00001, *I*^2^ = 84%) was noted, and the random effects model was used. The combined MD value and effect amount *Z* were 2.17 (95% CI: 1.15, 4.11) and 2.38 (*P* = 0.02), respectively. It showed that the risk of serum 25 (OH) D deficiency in AD patients was significantly higher than that in healthy controls (Figure 4).

The article "Serum Vitamin D Level and Efficacy of Vitamin D Supplementation in Children with Atopic Dermatitis: A Systematic Review and Meta-analysis" was published in 2022. Journal: Comput Math Methods Med.

### 3.4. Comparison of Serum 25 (OH) D Levels in Patients with Mild and Severe AD Rated by SCORAD Index

Serum 25 (OH) D levels in AD patients with mild and severe SCORAD index ratings were compared in 9 studies that included a total of 224 patients with mild AD and 196 with severe AD. The combined MD value and effect amount *Z* calculated by the random effects model was 9.23 (95% CI: 6.92, 11.55) and 7.82 (*P* < 0.001), respectively. The level of serum 25 (OH) D in patients with mild AD was significantly higher than that in patients with severe AD (Figure 5).

### 3.5. Comparison of SCORAD Scores of Pediatric AD Patients before and after Vitamin D Intervention

The SCORAD score at baseline and after vitamin D treatment in pediatric AD patients was evaluated in 5 studies that included 2 self-control experiments (Table 3). Given that the results of these two reports cannot be statistically integrated with the other 3 RCTs, subgroup analyses were performed. In total, 57 pediatric AD patients received vitamin D treatment in these 2 studies. There was no significant interstudy heterogeneity (*P* = 0.48, *I*^2^ = 0%), for which the fixed effects model was adopted. The combined MD and effect amount *Z* value were -18.80 (95% CI: -23.18, -14.42) and 8.40 (*P* < 0.001), respectively. The SCORAD scores decreased significantly by 18.8 points after vitamin D treatment in the self-control experiment (Figure 6). For the 3 RCTs, 47 AD patients received vitamin D supplementation. The fixed effects model is adopted. The combined MD and effect amount *Z* value measured by the fixed effects model (*P* = 0.23, *I*^2^ = 31%) were -11.02 (95% CI: -12.63, -9.40) and 13.34 (*P* < 0.001), respectively. The SCORAD score was significantly reduced by 11.02 points after vitamin D treatment (Figure 6). Although the number of studies is small, all studies demonstrated reduced SCORAD and improved clinical symptoms after vitamin D supplementation.

### 3.6. Effect of Vitamin D Supplementation on EASI Score

Three RCTs evaluated the effect of vitamin D intervention on EASI scores in patients with clinical AD. Study characteristics are summarized in Table 3. A total of 107 AD patients received vitamin D treatment, and 97 AD patients received placebo treatment. There was no significant heterogeneity among the literature (*P* = 0.78, *I*2 = 0%). The fixed effects model was adopted. The combined MD value was -3.72 (95% CI: -6.25, -1.19), and the combined effect amount was *Z* = 2.88 (*P* = 0.004). After vitamin D treatment, the EASI score of AD patients was significantly lower than that of the placebo treatment group by 3.72 points (Figure 7). Begg's test (Figure 8) showed no publication bias.

The article "Serum Vitamin D Level and Efficacy of Vitamin D Supplementation in Children with Atopic Dermatitis: A Systematic Review and Meta-analysis" was published in 2022. Journal: Comput Math Methods Med.

## 4. Discussion

This study comprehensively reviewed and summarized the results of case-control studies and interventional studies. Although it is found that the number of research literature is significant in the preliminary screening, the study quality varied significantly. Therefore, this study only included RCTs with a modified Jadad scale score ≥ 4 or case-control studies with a NOS ≥ 7. The results showed that the serum 25 (OH) D level of AD patients was significantly lower than that of the healthy control group. In addition, serum 25 (OH) D level in patients with severe AD was significantly lower than in patients with mild AD as indicated by the SCORAD. These results suggest that children with AD have a high risk of vitamin D deficiency. Studies have shown that [38] all individuals with vitamin D deficiency should receive serum 25 (OH) D monitoring regularly [13, 39]. Considering the higher risk of vitamin D deficiency in AD patients, vitamin D supplementation in this patient population can be considered in clinical practice.

Emerging studies have shown that the pathogenesis of AD is complicated that included destruction or weakening of epidermal defense barrier, immune dysfunction and gene susceptibility (such as silk protein gene deletion). In addition, allergens and microorganisms are also widely involved in the pathogenesis of AD due to skin barrier defects and innate immune system disorders [40, 41]. Although the exact relationship between vitamin D deficiency and AD remains incompletely understood, previous studies have shown that vitamin D deficiency may be involved in the occurrence and development of AD. Studies have shown that after vitamin D supplementation, antimicrobial peptides such as catheterin or *β*-defensin levels increased [42]. After the destruction of the vitamin D receptor, the levels of skin barrier proteins such as outer skin protein and silk fibroin decreased [43]. When the vitamin D level is low, the risk of higher IgE level and fixed value of Staphylococcus aureus in the population increases, while the level of interleukin-37 in the stratum corneum increases fourfold after vitamin D supplementation and reduces the occurrence of herpetic eczema [44]. These reports suggested that vitamin D can regulate immune response and maintain a healthy skin barrier function.

Our systematic review and meta-analysis that included recent high-quality studies is the latest research on the role of vitamin D in children with AD. This study found that the serum 25 (OH) D level of AD patients was lower than that of the healthy control group, and this reduction was statistically significant. In addition, we also supplemented the relationship between vitamin D deficiency, and patients with AD were more prone to vitamin D deficiency, which has not been mentioned in previous meta-analyses [9]. Due to the difference in sunlight exposure or latitude in various regions, the baseline vitamin D level in different areas varied dramatically. The relatively low vitamin D level does not necessarily mean vitamin D deficiency. This also explains the large heterogeneity with regard to vitamin D levels reported in this study. This study also confirmed that patients with AD have a higher risk of vitamin D deficiency and need continuous monitoring and vitamin D supplementation. The observation that serum 25 (OH) D level in severe AD patients was significantly lower than that of mild AD patients, indicating the decrease in vitamin D level and deficiency may be related to the aggravation of AD.

The article "Serum Vitamin D Level and Efficacy of Vitamin D Supplementation in Children with Atopic Dermatitis: A Systematic Review and Meta-analysis" was published in 2022. Journal: Comput Math Methods Med.

Self-control experiments and RCTs included in this study showed the improvement of SCORAD and EASI score after vitamin D supplementation. Therefore, vitamin D supplementation is beneficial to AD patients. However, the number of included studies is small, and the interpretation of the results needs to be more cautious. In addition, differences in vitamin D levels during seasonal and latitudinal changes also affect the evaluation of vitamin D supplementation. Moreover, the dose and duration of vitamin D used in different studies vary greatly with many confounding factors that prevented from exploring real impact of vitamin D supplements on children. More large-scale prospective RCT studies with different vitamin D supplement doses and duration are needed to obtain adequate treatment options.

The literatures included in our study are high-quality studies, which is the advantage of this study. Similar literatures have recently compared the effects and efficacy of serum vitamin D levels and vitamin D supplementation on children with AD [45] with similar conclusions. However, we focused on pediatric AD, whereas other studies often presented mixed patient population that included both children and adults. Factors like age create considerable interstudy heterogeneity and reduce the confidence and clinical generalizability of the results. In addition, the evaluation indicators of other studies were single with only the SCORAD score used to evaluate the effect of vitamin D supplementation. In our study, the two indicators are used for comparison, and more reports are included in the evaluation, making the results more credible. Of note, there are many confounding factors in vitamin D research, such as the latitude, the time of sunlight exposure, and the type, dose, and duration of vitamin D supplements. Due to the wide heterogeneity and lack of homogeneous researches, these potential confounding factors were not considered. This also suggests that a larger sample, multicenter or prospective, highly homogeneous RCTs or cohort studies need to be carried out. A more reasonable and unified result analysis system should be adopted to provide higher-level evidence.

The article "Serum Vitamin D Level and Efficacy of Vitamin D Supplementation in Children with Atopic Dermatitis: A Systematic Review and Meta-analysis" was published in 2022. Journal: Comput Math Methods Med.

In conclusion, this study systematically summarized and analyzed the evidence of the interaction between vitamin D and children with AD. It showed lower serum 25 (OH) D level and increased risk of vitamin D deficiency in pediatric AD patients as compared with healthy controls. The serum 25 (OH) D level in severe AD patients was significantly lower than that in the mild AD patients. The SCORAD and EASI score improved after vitamin D supplementation, suggesting its beneficial effect to AD patients. At the same time, more homogeneous studies are needed to reduce confounding factors and further evaluate the impact of vitamin D treatment on the outcome of AD patients.

## Figures and Tables

**Figure 1:** Flow chart of literature screening.

**Figure 2:** Risk assessment of bias in randomized controlled trials.

**Figure 3:** Comparison of serum 25 (OH) D levels between AD patients and healthy controls.

**Figure 4:** Comparative meta-analysis of serum 25 (OH) D deficiency between AD patients and healthy controls.

**Figure 5:** Comparative meta-analysis of serum 25 (OH) D levels in AD patients with mild and severe SCORAD index rating.

**Figure 6:** Meta-analysis of SCORAD scores of clinical AD patients before and after vitamin D intervention experiment.

**Figure 7:** Comparative meta-analysis of the effect of vitamin D intervention experiment on EASI score of clinical AD patients.

**Figure 8:** Comparative meta-analysis funnel chart of the effect of vitamin D intervention experiment on EASI score of clinical AD patients.

**Table 1:** Basic characteristics and document quality scores of included documents.

Study	Study design	Studies assessment scale
Lipińska, 2021	CCT	7
Ahmed, 2021	CCT	8
Sanmartin, 2020	CCT	7
Raj, 2020	CCT	7
Xiang, 2019	CCT	7
Lee, 2019	CCT	8
Daniluk, 2019	CCT	8
Machura, 2018	CCT	7
Dogru, 2018	CCT	7
Su, 2017	CCT	8
D'Auria, 2017	CCT	9
Sharma, 2017	CCT	7
Cheon, 2015	CCT	8
Di Filippo, 2015	CCT	7
Wang, 2014	CCT	7
El Taieb, 2013	CCT	7
Lara, 2019	RCT	5
Amestejani, 2012	RCT	6
Javanbakht, 2011	RCT	6
Camargo, 2014	RCT	4
Mansour, 2020	RCT	6
Sidbury, 2008	RCT	5

RCT: randomized controlled trial; CCT: controlled clinical trial; studies' assessment scale: RCT study uses the modified Jadad scale; CCT study uses Newcastle-Ottawa scale.

The article "Serum Vitamin D Level and Efficacy of Vitamin D Supplementation in Children with Atopic Dermatitis: A Systematic Review and Meta-analysis" was published in 2022. Journal: Comput Math Methods Med.

**Table 2:** Characteristics of included studies on serum 25 (OH) D level between AD patients and healthy controls.

Study	Year	Study population age (AD group/control group) (years)	Study size	Location
Lipińska et al.	2021	Median age (7/8)	75 cases, 37control subjects	Poland
Ahmed et al.	2021	Mean age (11/9.2)	100 cases, 101 control subjects	Egypt
Sanmartin et al.	2020	Age range (0-12/0-12)	134 cases, 105 control subjects	Spain
Xiang et al.	2019	Mean age (5.1/3.2)	81 cases, 65 control subjects	China
Lee et al.	2019	Mean age (8.6/9.4)	135 cases, 65 control subjects	Malaysia
Daniluk et al.	2019	Median age (6/5.5)	29 cases, 22 control subjects	Poland
Machura et al.	2018	Age range (2-14/2-14)	57 cases, 34 control subjects	Poland
Dogru et al.	2018	Mean age (5.6/5.4)	69 cases, 70 control subjects	Turkey
Su et al.	2017	Mean age (6.5/7.4)	60 cases, 37 control subjects	Turkey
D'Auria et al.	2017	Mean age (6.2/6.1)	52 cases, 43 control subjects	Italy
Sharma et al.	2017	Mean age (6.1/6.7)	40 cases, 40 control subjects	India
Cheon et al.	2015	Median age (6/6)	91 cases, 32 control subjects	Korea
Wang et al.	2014	Median age (6/5.5)	498 cases, 328 control subjects	Hong Kong
El Taieb et al.	2013	Mean age (6.1/6.5)	29 cases, 30 control subjects	Egypt

**Table 3:** Summary of characteristics of intervention experiments included in the study.

Study	Year	Study design	Study size	Duration	Dose/daily	Location	AD severity assessment
Raj et al.	2020	RMI	35 cases	3 months	1000 IU	India	SCORAD
Di Filippo et al.	2015	RMI	22 cases	3 months	1000 IU	Italy	SCORAD
Lara et al.	2019	RCT	11 cases, 24 placebos	3 months	1000 IU	Canada	SCORAD
Amestejani et al.	2012	RCT	11 cases, 12 placebos	60 days	1600 IU	Iran	SCORAD
Javanbakht et al.	2011	RCT	24 cases, 26 placebos	60 days	1600 IU	Iran	SCORAD
Mansour et al.	2020	RCT	44 cases, 42 placebos	12 weeks	1600 IU	Egypt	EASI
Camargo et al.	2014	RCT	58 cases, 49 placebos	1 month	1000 IU	Mongolia	EASI
Sidbury et al.	2008	RCT	5 cases, 6 placebos	1 month	1000 IU	USA	EASI

RMI: repeated measure interventions (patients are their own control); RCT: randomized controlled trial; SCORAD: Scoring Atopic Dermatitis; EASI: eczema area and severity index.

## Data Availability

The data used to support the findings of this study are included within the article.
